# Intelligent Recognition Technology for the Segmentation of Traffic Indication Images Concerning Different Pavement Materials

This article has been retracted.

**DOI:** 10.1155/2022/6278240

**Published:** 2022-09-20

**Authors:** Juanhong Xie, Guojian Shi, Weizhi Zhu

**Affiliations:** Guangdong Technology College, Zhaoqing, 526100 Guangdong Province, China

## Abstract

Traffic indication is an important part of the road environment, providing information about road conditions, restrictions, prohibitions, warnings, and the current status related to the flow of the traffic and other navigational aspects. The shape, color, and pictogram of a traffic indication are encoded into the visual characteristics of traffic signs. Not paying attention to these traffic signs could lead directly or indirectly to traffic accidents. In this article, the support traffic indication vector recognition (STIVR) method is proposed to classify the best signal detection to avoid traffic congestion and accidents. The proposed STIVR recognizes the traffic indication system automatically, reduces occurrences of traffic accidents, and helps drivers move safely on different pavement materials. Besides, the adaptive median filter (AMF) algorithm is used to pre-process and protect the traffic indication images without obscuring them. Thus, it indicates the edge of the non-smoothed nasty ferment from the service. In the detection of traffic events, indication images are enhanced, pre-treated, and divided according to symbols and their characteristics such as color, shape, or both. The output becomes a segmented image, including the available space identified as a road sign. The experimental results show that the proposed method functions well; achieves a sufficiently higher process speed and better segmentation of traffic indications and more accuracy in recognition of the objects. For example, the proposed method reaches a higher sensitivity performance of 96%.

## 1. Introduction

Across the globe, important information about the speed limits and road conditions needs to be given visually to drivers such as traffic indications and lane information. Its purpose is to recognize and detect traffic indications easily based on their color or shapes. The traffic indication symbol carries a lot of useful information. It is operated when the vehicle turns, for example, to the right lane by suggesting the appropriate speed to the driver. To avoid obstacles and potential risks, inform the current network issues related to the network of the traffic, road and lane conditions, location information, and other vehicles' driving information, so they are significant to protect both drivers and pedestrians. Thus, the traffic right to securely travel is guaranteed for all parties. For instance, this kind of system could help blind pedestrians as well as assist advanced drivers too. Therefore, operators do not have to check signs regularly.

Figure 1 defines the well-known traffic indications seen by travelers by car or by foot. Their shapes and colors are different. Most of these traffic indicators can be understood easily. The purpose of this task is to classify various road traffic indications automatically by an algorithm. When any algorithm is used for this purpose to detect and recognize traffic signs, it is expected that the proposed algorithm should work and function in any environment as versatile as possible when a large set of road traffic indications are available. So, the main motivation is to apply this proposed algorithm to road signs of any country, any language, any color, and all types of traffic networks. Therefore, the five shapes (circle, triangle, square, pentagonal, or octagonal) should be detected and recognized to cover a general framework as a reference database.

Weather conditions such as cloudy, rainy, snowy, foggy, and so on should be detected in different geographic, climatic, and landscape situations. For example, the variable called lighting conditions could occur uncontrollably on any given day, e.g., the Broadway light and sunset times. To resolve the issues mentioned above, a new traffic sign is needed to be proposed that could function with a high success rate. However, there exist challenges to detect well-known traffic indications due to auxiliary color, shape, size, and location of signs. Under normal circumstances, the symbol could occasionally be tilted, but detection will be constantly rotating, zooming, and panning, standing next to the road. Furthermore, the system is expected to be robust in partially clogged situations and under various lighting conditions.

The rest of the paper is constructed as follows: Section 2 presents the related work. Section 3 is allocated to the proposed method. Section 4 presents the results of the proposed method. The discussion is provided in Section 5. Section 6 concludes the research.

## 2. The Related Work

The convolutional neural network (CNN) can be utilized not only for the image data sets but also employs metadata in the form of heterogeneous deep data sets [1] and could assign all of the traffic light information related to the lane information system. To accomplish this, the general CNN topology is trained by converting the input images to predict down-sampling data sets and index vectors [2]. Displaying locations associated with the channel vector contain all the associated traffic light columns. Then, adaptive weighting features of the metadata are simultaneously ready to convolute with a convolution layer that is the characteristic of the selected input mapping and mapping fusion [3].

Both recognition and automatic detection of traffic signs play an important role in managing the inventory of traffic signs [4]. This system provides an accurate and timely tool to manage the inventory of traffic signs with minimum human effort. In computer vision systems, the detection of traffic signs and recognition of community-related issues grows significantly [5]. The most readily available methods for the assistance system of advanced drivers and automatic detection of traffic signs are needed to work on.

The high-performance traffic sign recognition (TSR) framework can be conducted by detecting various traffic signs in rapid high-resolution images [6]. The framework consists of three parts: the new region extraction method concerning the extraction of high-contrast regions, cascading tree detectors, and fast shutdown robust stream based on the classification of all sparse representations of extensions [7]. Unlike color threshold or pre-processing terminal region, region-of-interest (ROI) extraction allows a good balance between the extraction rate and the detection rate as well as a high local contrast [8].

The recognition of traffic signs plays an important role in the operation of the support system and intelligent autonomous vehicle system. Real-time performance, in addition to its recognition performance, grows ideally [9]. To resolve issues related to various traffic signs, image processing of the speed input shows the real-time sign recognition of a traffic area. To achieve this goal, a detection module is firstly proposed, which is the best available detection module, that works efficiently when the speed of the vehicles is 20 times faster [10].

The potential data type for the placement and location codes provided by a system having traffic signs are associated with the inspection process space. To obtain a movement of the laser scanning, the traffic sign presents inventory application such as scene points on the traffic sign whose reflective properties are related to the algorithm when the detection of the complex road conditions are under consideration [11–12].

The image registration of processing point groups was proposed to highlight a group of traffic signs on the two-dimensional image plane [13]. The third dimension, according to the extracted traffic sign point, creates a relationship between the geospatial traffic signs and the road environment, thus recommending a process to check the location of the traffic signs and layout [14, 15].

Simultaneously, the detection system of the new traffic sign determines the exact boundaries of traffic signs and their location and estimates it by using a CNN [16]. Therefore, the traffic sign can estimate the exact boundaries of the road environment, so a smart car navigation system is essential to function. Before including the recent CNN method, the detection system of the traffic sign provides a boundary traffic sign box as the only output to estimate contour or image segmentation. Hence, additional processing is needed to obtain the correct boundaries of the code [17].

Two symbols and signs are employed to detect and classify text focusing on the most common European cities. The system consists of three phases: traffic sign detection, purification, and classification [18]. The method that marks a 164-pixel extended version of the German Traffic Sign Detection Benchmark (GTSDB) is divided into eight categories [19].

High-speed and high-definition images detect traffic signs, and the accuracy of recognition increases the traffic image's different areas of interest [20]. Each traffic image in the convolution neural network determines these regions after applying graphical and parallel detection and recognition by utilizing efficient and parallel pre-processing means. More recent research related to the motivation of the manuscript can be found in references [21, 22].

## 3. The Proposed Method

Recognition and automatic detection of road traffic indications are used to adjust the important tasks to warn and guide drivers and pedestrians. The first step of the AMF algorithm is based on pre-processing data by removing noises, then feature extraction by using the Fourier descriptor technique is implemented, thirdly processing of image segmentation of traffic indication shapes and colors using the dynamic threshold algorithm is conducted, and finally, the STIVR algorithm is used to identify the traffic indication. To detect and identify landmarks in traffic settings, several techniques have been developed within the scope of its application. The driver assistance system can detect and identify landmarks in real-time. So, it helps improve traffic flow and safety and avoid dangerous driving consequences such as collisions.

Figure 2 defines how the raw images of the traffic indication dataset are collected and pre-processed to remove noises; then, it presents feature extraction to select the best features. Finally, image segmentation is used to select the colors and shapes of the traffic indication images and classify the traffic detection.

### 3.1. The Dataset of the Raw Traffic Images

The image dataset is simply a collection of traffic indications that have been collected by the camera. The collected traffic signs under different lighting conditions, different weather conditions, and different image geometry concerning various lighting conditions may contain some drawbacks. Besides, they have different colors, shapes, and logos belonging to different categories, which can be seen under different conditions. Traffic images in the dataset, such as clogging damaged or faded, weather conditions, light, geometry, and the state of the sign, such as blurring due to defective image, are classified according to the code type. The number of traffic indication images containing the same type of signs should be extended to provide a good example of training. Accessing the dataset makes it possible to easily select an image with specific characteristics to manage the images and information of the traffic sign.

### 3.2. Pre-Processing of Traffic Indication Images Using Adaptive Median Filter (AMF)

The pre-processing of the traffic indication images is the first step for the proposed traffic indication system called the STIVR. The main purpose is to remove reflections, which are low-frequency background noise. Then, the image of each particle is normalized, which indicates the intensity for the important parts of the image using the AMF algorithm. The image within the input image is divided into separate channels R, G, and B. In the proposed method, the filter is applied to a threshold value for each channel to select the pixel value that falls within the range of the objective. Often the dataset of the traffic training image to search is based on the precise position of the pixel, and objects in the image that are represented binarily.

### 3.3. Feature Extraction of Traffic Indication Images for Using the Fourier Descriptor Technique

Feature extraction is described such that the pattern in the classification task is a formal process that is very easy to conduct pattern information related to the shape, which is called the process dealing with image pattern recognition of traffic signs wherein a special form of dimension reduction using the Fourier descriptor technique is implemented. The proposed transformation technique called the Fourier descriptor technique is widely used for feature extraction and shape analysis. The coefficients are used to form the shape descriptor, which indicates the shape of the frequency domain. While a lower frequency descriptor contains information regarding the general functions of the shapes, a higher frequency descriptor contains information about the finer detail shapes.

### 3.4. Segmentation of Traffic Indication Images Using the Dynamic Threshold Algorithm

The segmentation of the traffic indication images is an important step to eliminate all non-critical information regarding the background of the object images. It produces a binary indication image containing other objects in colors and shapes for road traffic signs. Because it reduces the number of basically possible objects, this step reduces the computational burden by using the dynamic threshold algorithm (DTA).

### 3.5. Classification of Traffic Indication Images Using Support Traffic Indication Vector Recognition (STIVR)

The proposed STIVR traffic indication posting the range of an area determines the system that can detect the distance of traffic signs. It has the same range of pixel values outside this range that cannot be a marking for the traffic. At this level, such a central area and the maximum width of each region's important information are calculated. The proposed STIVR algorithm is used to classify the traffic indication information. Then, each area will be used to determine whether it is a traffic sign or not. Afterward, the spot image of the detected traffic signs is passed to the STVIR for recognition purposes.

### 3.6. Algorithm

Begin

Stage 1: Import the traffic indication dataset

Stage 2: Separate dataset into train dataset and test dataset

Stage 3: Classify the traffic indication dataset

Stop

Figure 3defines the issues that are related to automatic detection of weather conditions such as cloudy, rainy, snowy, foggy, and so on in different geographic, climatic, and landscape conditions besides cluttered background and foreground landscapes in the current road traffic indicators. For instance, the variable called lighting conditions could occur uncontrollably on some days, e.g., the broadways light and sunset times.

## 4. Results

Recognition technology and automatic detection of road traffic signs are conducted by the proposed method called STIVR. The traffic indications in road networks are used to adjust warnings and guidance that drivers and pedestrians face.

Table 1 defines the evolution of parameters in the proposed algorithm called STIVR. The literature contains other algorithms such as CNN and GTSDB.

Table 2 identifies the performance of the STIVR based on the classification of indications by using the criteria called specificity and sensitivity. The proposed algorithm outperforms others available in the literature.

Figure 4 identifies the classification performance of traffic indications. The proposed method called STIVR provides a 96% success rate that is much higher than those of the CNN, which is 60%, and the GTSDB, which is 55%.

Figure 5identifies the specificity and sensitivity that correctly defines the traffic indications of the specific conditions and correctly defines unrelated ones. STIVR algorithm provides a specificity result of 96%, which is much higher than those of the CNN, which is 50%, and the GTSDB, which is 45%.

Figure 6 depicts the evolution of sensitivity performance of the proposed method that reaches 96% sensitivity. The result is much better than those of the CNN, which is 50%, and the GTSDB, which is 45%.

Figure 7 depicts the evolution of false rate performance with more accurate outcomes and real-time detection of traffic signs that have a lower false rate, which is very essential to improve road safety and driving efficiency. The STIVR algorithm provides a 96% false rate. It is much better than those of the neural network (CNN), which is a 60% false rate, and the GTSDB, which is a 65% false rate.

## 5. Discussion

The proposed algorithm, called the STIVR, has better performance when compared with other algorithms available in the literature. The advantages of the proposed method can be summarized as follows:

(a) It has a 96% success rate in the classification performance of traffic indications.

(b) It has a 96% specificity results.

(c) It reaches 96% sensitivity outcomes.

(d) It provides a 96% false rate.

## 6. Conclusion

Traffic sign detection is the most important phase in the process of traffic sign indication. A method called the STIVR is proposed to classify the traffic indications by combining information on color or shape features or both. The proposed traffic image identification method utilizes both similarity and shape measurement that can achieve a better detection outcome having better sensitivity, specificity, and false rates. Besides, the proposed adaptive median filter is used for pre-processing the data sets. Moreover, the Fourier descriptor technique is used to conduct the feature selection process, and the dynamic threshold algorithm is used for the traffic image segmentation process. The proposed STIVR algorithm is used to finally classify the best traffic indication outcomes with higher sensitivity and specificity outcomes.

## Figures and Tables

**Figure 1:** Traffic indications [1]. Source: https://civilnoteppt.com/traffic-signs-or-road-signs-in-india/.

**Figure 2:** The proposed diagram of the traffic indication.

**Figure 3:** The circuit diagram for the detection of the traffic indications.

**Figure 4:** The performance of the traffic indication.

**Figure 5:** The evolution of the specificity performance.

**Figure 6:** The evolution of the sensitivity performance.

**Figure 7:** The evolution of the false rate performance.

**Table 1:** Evolution of parameters.

Parameters	Values
Tool	Anaconda
Language	Python
Name of dataset	Traffic indication dataset
Number of datasets	300
Training dataset	250
Testing dataset	50

**Table 2:** The analysis of the proposed method.

No of data	Performance of traffic indication classification			Specificity performance			Sensitivity performance		
	CNN in %	GTSDB in %	STIVR in %	CNN in %	GTSDB in %	STIVR in %	CNN in %	GTSDB in %	STIVR in %
1	75	70	80	65	60	80	60	65	82
2	70	65	85	60	55	87	55	60	89
3	65	60	90	55	50	92	50	55	92
4	60	55	96	50	45	95	45	50	96

## Data Availability

Data will be provided upon request to the authors.
